The article "Why Mechanism Matters: A Literature Review of Simultaneous Ipsilateral Tibial Tuberosity Avulsion and Patella Fracture With Case Report" was published in 2021. Journal: Cureus.

# Why Mechanism Matters: A Literature Review of Simultaneous Ipsilateral Tibial Tuberosity Avulsion and Patella Fracture With Case Report

**DOI:** 10.7759/cureus.20232

**Published:** 2021-12-07

**Authors:** Joseph Muscat, Aroon Baskaradas, Govind Dhillon, Vashist Motkur, Raj Thakrar

**Affiliations:** 1 Trauma and Orthopaedics, East and North Hertfordshire Trust, Stevenage, GBR; 2 Orthopaedics and Trauma, Royal Surrey County Hospital, Guildford, GBR

**Keywords:** unilateral and extensor mechanism disruption, ipsilateral, bifocal, tibial tuberosity avulsion, patella

## Abstract

Simultaneous ipsilateral tibial tuberosity avulsion and patella fractures are rare in adults. They are often associated with patients who have underlying bone disease and other medical co-morbidities. Here we describe a case where this injury was attributed to direct trauma and demonstrate our department’s management for such an injury. In addition to our case report, we have performed a systematic literature review to identify other cases of the same injury. Only four other cases have been reported. Here we summarise and compare the management and outcome measures reported in each case.

All patients are managed differently, yet all authors report satisfactory outcomes. With this being a relatively rare injury, further research is required to establish a gold standard for management of such patients.

## Introduction

Tibial tuberosity fractures are more typically seen in the paediatric and adolescent population, particularly in athletic male adolescents approaching skeletal maturity [1]. In the adult population these fractures are rare [2]. Patellar fractures are complex injuries that impact mobility due to disruption of the extensor mechanism. There are favourable outcomes for function in patients that are selected for operative management [3]. Knee injuries commonly result in injury of the extensor mechanism, it is key for a gait, stability and activity of daily living [4]. A crucial part of the extensor mechanism is formed by the patellar tendon which originates from the patella inferior pole and then inserts tibial tuberosity [4]. The extensor mechanism is based on dynamic and static forces centred around the patellar and its tendinous insertion into the tibial tuberosity [5]. When the extensor mechanism is repaired there are significantly higher rates of adverse outcomes if they are mobilised early, however, prolonged immobilisation contributes to decline of mobility, decreased quality of life and increased financial burden [6]. Studies on patellar fractures have estimated that approximately 10 weeks would be required to achieve bony healing if patients were able to mobilise early, which puts a high workload on any surgical fixation [7].

Extensor mechanism disruption can occur in a variety of patterns to injuries in combination of the patella, patella ligament and tibial tubercle. Cases of bifocal extensor mechanism disruption are rare, particularly those which involve a fracture of both the patella and tibial tuberosity [8]. Kang et al. have previously described a case of simultaneous ipsilateral tibial tuberosity avulsion and patella fracture in an elderly male patient. They proposed a classification system for types of extensor mechanism disruption with the type 4 pattern described as “*avulsion fracture of the tibial tubercle with avulsion fracture of the inferior pole of the patella*” [8]. A summary of their classification system is shown below:

Type 1: avulsion fracture of the tibial tubercle with avulsion of the patella ligament from the tibial tubercle;

Type 2: avulsion fracture of the inferior pole of the patella with avulsion of the patella ligament from the tibial tubercle;

Type 3: avulsion fracture of the tibial tubercle with rupture of the quadriceps tendon;

Type 4: avulsion fracture of the tibial tubercle with avulsion fracture of the inferior pole of the patella;

Type 5: rupture of the quadriceps tendon with avulsion of the patella tendon from the patella

Given the unique injury and significant impact on extensor mechanism and mobility, it is important that further research is done to collate these cases and compare management and outcomes. In this paper, we focus on type 4 injuries as proposed by Kang et al., we have performed a literature review on reported cases of simultaneous ipsilateral tibial tuberosity and patella fractures in adults, in addition to presenting our own case report of a patient seen and managed in our unit.

## Case presentation

We present a case of a 70-year-old female. She was outdoors in a wooded area and fell from standing onto uneven hard surfaces (see Figure 1) with a flexed knee and suffered an injury to her knee area. On examination, there was tenderness over the patella and tibial tuberosity. She was unable to bear weight due to pain but able to perform a straight leg raise. It was a closed, neurovascular intact injury. There was a small abrasion to her nose, but no other injury was noted. Her past medical history included mild depression, for which she was taking fluoxetine. She was independent and walked up to 10 km a day prior to the injury. She was a non-smoker and did not drink alcohol.

 

**Figure 1:** Picture illustrating the mechanism of injury. The patient had tripped on a tree root (red arrow) and directly impacted her patella and proximal tibia on two rocks (blue arrows).

Upon questioning, the patient reported the unique nature of her fall and provided our Orthopaedic team a photograph taken on her mobile phone of the site of injury. It appears that the patient tripped on a tree root (Figure 1 red arrow) and directly impacted her patella and proximal tibia on two rocks (Figure 1 blue arrows).

The X-ray images of the patient’s left knee that were taken in the emergency department are shown in Figure 2. The patient sustained a minimally displaced tibial tuberosity fracture. A CT scan was subsequently obtained and key images are displayed in Figure 3. They demonstrated a vertical oblique fracture extending superiorly to the tibial plateau, breeching the cortex in the region of the intercondylar notch. There was a 6 mm depressed fragment of the lateral condyle. In addition, there was a minimally displaced transverse fracture of the inferior patellar, extending to the patellar tendon origin with minimal comminution.

**Figure 2:** Pre-operative anterior-posterior (A) and lateral (B) radiographs taken in the emergency department.

**Figure 3:** Axial (A,B), sagittal (C) and coronal (D) images of pre-operative CT scan of the left knee.

The patient was admitted and operated on 48 hours after the time of injury. She underwent an open reduction and internal fixation. Intraoperative images are shown in Figure 4. The operation was done under spinal anaesthetic with a leg tourniquet. The approach to the tibia was through two stab incisions. Two partially threaded tibial screws with washers were used to achieve compression. The patella was approached through a midline incision, two K-wires were inserted in parallel and two partially threaded screws were used with a tension band wire to achieve reduction.

**Figure 4:** Lateral (A,B) and anterior-posterior (C) radiographs taken intra-operatively.

The patient was discharged 24 hours post-operation, with a hinged knee brace (0-30 degrees of flexion) and instructions to partial weight bear for 6 weeks. She was followed up 2 and 6 weeks post-operatively. At 6 weeks, her range of motion was 0-90 degrees and there were no postoperative complications. Radiographs taken at 6 weeks are shown in Figure 5. She could fully bear weight without pain. She was discharged from the fracture clinic, but continued physiotherapy for ongoing rehabilitation. Documented consent was obtained for all photographs and images.

**Figure 5:** Lateral (A) and anterior-posterior (B) radiographs taken six weeks post-operation.

## Discussion

Literature review-Methodology

Search Strategy

A systematic search was conducted in accordance with the Preferred Reporting Items for Systematic Reviews and Meta-analyses (PRISMA) guidelines on Covidence software (Covidence systematic review software, Veritas Health Innovation, Melbourne, Australia. Available at www.covidence.org) [9].

We systematically searched PubMed databases using Key words such as tibia, patella, fracture, tibial tuberosity avulsion, bifocal, ipsilateral, unilateral, extensor mechanism disruption, used in combination with Boolean terms-AND, OR. A parallel search was also conducted by library staff of Medline and Embase databases. We aimed to identify cases that reported ipsilateral tibial tuberosity avulsion and patella fracture in adults.

Inclusion Criteria

Eligible cases for inclusion satisfied the following criteria: 1) Adult humans (>18 years); 2) ipsilateral tibial tuberosity avulsion and patella fracture (type 4 extensor mechanism injury); 3) fracture of both bones; 4) patient management included, 5) patient outcome reported.

Exclusion Criteria

Studies were excluded for the following criteria: 1) cadaveric; 2) animal study; 3) paediatric cases (<=18 years); 3) biomechanical studies; 4) single bone fracture; 5) soft tissue injury only; 6) morphology studies; 7) simulation studies.

Screening

Titles and abstracts were screened using the Covidence software by authors (JM and GD) independently. Where eligibility was unclear, the full text was retrieved and assessed. Disagreements were resolved by discussion.

Data Analysis

Data collected was independent of other cases, with varied information, they have not been collated before. Descriptive analysis was performed on our results, we analysed the data available and presented it as values shown as percentages (%) or total number (n).

Results

Our search identified 528 articles, after screening eight were selected for full-text review and that produced four cases, including the Kang et al.’s case (five cases in total were included for the final comparison, they included our patient, and four other case reports from the literature search). They all fit the type 4 pattern of injury-avulsion fracture of the tibial tubercle with an avulsion fracture of the inferior pole of the patella. Please see Figure 6 for the full PRISMA flowchart.

**Figure 6:** Prisma flowchart showing cases reviewed and included for analysis.

60% (3/5) of the patients were male, 20% (2/5) were female. The mean average age of all patients was 74.4 years, the average age for females was 70 years old and males was 70.66 years old. Two of the five patients (40%) had a form of mental health disorder (psychosis and depression), two of the five had previous osteoarthritis (40%). The mechanism of injury was the same in four/five cases (80%)-falling onto flexed knees. There was one case of a patient sustaining a twisting injury. Choices of surgical management varied between the cases. The choices of patella fixation included-tension band wire, suture fixation, no fixation, and two cases had a combination of vertical screws/pins and tension band wiring. The tibial tuberosity method of fixation included two cases of tension band fixation and three cases of cannulated screws. The combination of choice of fixation for the patella and tibial tuberosity varied between all cases. One case required fixation of the patella tendon.

Postoperative instructions varied, three/five were put into a cylindrical cast. One patient was put in an extension splint and one in a hinged knee brace. Two/five were allowed for full weight-bearing, two/five were allowed for partial/touch weight-bearing and one patient was not allowed to bear any weight. All were given varying degrees of range of motion, with some being permitted to have a full active range (2/5) of motion and others (3/5) having a passive range of motion.

Length of follow-up ranged from two to 46 months, one required removal of metalwork at 17 months post-index procedure, one reported 20 degrees of extensor lag. There was no report of any significant adverse outcomes in each of the reports. The cases are summarised in Table 1.

Discussion

The proposed mechanism for such an injury pattern has been thought to occur through one of two mechanisms. One mechanism is via a direct blow to both the patella and tibial tuberosity. The other by direct force to the patella tendon, resulting in forces being transmitted to both the proximal and distal tendon, resulting in fractures of both the origin and insertion [10].

Chautems et al. [11] were the first to report on such a double bony avulsion fracture in an adult. The mechanism of injury was a fall onto the knee in a 90-year-old female. Concurrent opposing forces on the ligament in the context of osteoporotic bone quality were described as the cause of the bifocal disruption. This paper required translation into English.

Yoon et al. [12] described a case in a 50-year-old who sustained an avulsion fracture of the patella and tibial tuberosity in an ectopic ossified patella tendon following a twisting injury. They suggest that the geometry of the fracture pattern could be related to the ectopic ossified patella tendon.

Kang et al.’s [8] case was that of an 84-year-old male who was involved in a motorcycle accident. They also attribute the injury pattern to a direct force onto the patella tendon in a highly flexed knee, resulting in force to both the proximal and distal parts of the tendon, which led to the avulsion fractures. More recently, MacDonald et al. [13] also describe a case of a type 4 injury in a 56-year-old male, who also fell onto a flexed knee. They suggest that poor bone quality, due to smoking and antipsychotic medication history, attributed to the injury pattern.

Our patient was relatively young and still very active, with no previously documented bone or knee pathology. It was noted that the patient was taking fluoxetine. Several studies have demonstrated an association between antidepressant use and bone loss in post-menopausal women [10,14]. This certainly could have been an attributing factor, given the low energy mechanism of injury. When stress is applied to the patella tendon, this increases strain at the bone-tendon interface of the tendon origin and insertion and can result in an avulsion fracture, particularly in poor bone [13]. However, in our patient, there was clear evidence from the mechanism described by the patient of direct force being applied to both the patella and tibial tuberosity, rather than contraction of the patella tendon resulting in avulsions. Our patient’s fracture pattern was more severe than those previously described, including comminution of the patella, in addition to intraarticular extension of the tibial plateau. As noted, different management strategies were employed in each case, but all reported satisfactory outcomes. The cases are summarised in Table 1.

**Table 1:** Summary of cases included in the study. PMH: past medical history

Author	Patient (Age)	PMH	Mechanism of injury	Fixation method	Post operative instructions	Outcome
Chautems et al. 2001 [11]	Female (90)	Diabetic—non-insulin -dependent, mild osteoarthritis	Fall onto flexed knee	Patella: two vertical pins and figure-of-eight cerclage. Tibial tuberosity: three staples and cerclage wire	Loading under extension splint protection from Day 4. Passive flexion limited to 60 degrees from Day 8 until bone consolidation	No complication reported. Patient was walking at 6 months with the aid of two sticks
Yoon et al. 2007 [12]	Male (72)	Osteoarthritis in both knees. Previous right-sided femur fracture 50 years ago	Twisting injury to knee	Patella: tension band wire Tibial tuberosity: tension band wire. Patella tendon: fixed with absorbable sutures	Immobilised in full extension cylindrical plaster cast with full weight-bearing for several weeks, then passive range of motion exercises	Required removal of metalwork at 17 months. At 46 months, no functional impairment and radiological signs of bony union
Kang et al. 2013 [8]	Male (84)	Hypertension	Fall onto flexed knee	Patella: suture fixation Tibial tuberosity: cannulated screws	Long leg cast for 6 weeks and non-weight-bearing. Then commenced partial weight-bearing and active range of motion in the knee	Follow-up at 2 months showed bony union of the tibia, but 2 mm displacement of the patella. There was 20 degrees of extensor lag. At 12 months, there was radiological union of the patella, full range of motion in the knee and a Saltzman patellofemoral score of 92 (excellent)
MacDonald et al. 2021 [13]	Male (56)	Autism, psychosis, long-term smoker	Fall onto flexed knee	Patella: no fixation. Tibial tuberosity: cannulated screws	Cylinder cast for 2 weeks, and later hinged knee brace following, increasing the range of flexion every 2 weeks. Toe-touch weight-bearing for the first 4 weeks, then progressively allowed to increase weight-bearing status	Walking comfortably at 8 weeks without aids and full range of motion in the knee. At 1 year, back to full activity
Author’s case	Female (70)	Mild depression	Fall onto flexed knee—direct impact to the patella and tibia	Patella: vertical screws and tension band wire. Tibial tuberosity: cannulated screws	Hinged knee brace and partial weight-bearing for 6 weeks	At 6 weeks her range of motion in the knee was 0-90 degrees and she could bear weight fully with no aids. Discharged from clinic

## Conclusions

Given the limited reports of such injuries, common protocols for the management in adults do not exist. Our case demonstrates that open reduction and internal fixation of both the tibial tuberosity and patella fracture, with partial weight-bearing and restricted knee flexion can produce a satisfactory outcome. These types of injuries are rare. One should always consider underlying bone pathology and contributing medical co-morbidities when assessing the patient. Understanding the mechanism of exactly how the patient fell can help understand how such an injury may have been sustained. Open reduction and internal fixation of both the tibial tuberosity and patella, with partial weight-bearing and reduced knee flexion is one potential management strategy for such an injury. Further research is required to further establish a recommended treatment method based on comparable outcomes.
